# Transcriptome Comparison of Brain and Kidney Endothelial Cells in Homeostasis

This article has been retracted.

**DOI:** 10.1155/2022/5239255

**Published:** 2022-01-28

**Authors:** Xiaohua Huang, Zhongshi Huang, Zhongheng Wei, Yun Feng, Xuebin Li, Anding Xu, Chongdong Jian

**Affiliations:** ^1^Jinan University, Guangzhou, Guangdong Province, China; ^2^Department of Neurology, The Affiliated Hospital of Youjiang Medical University for Nationalities, Baise, Guangxi Province, China; ^3^Center for Systemic Inflammation Research, School of Preclinical Medicine, Youjiang Medical University for Nationalities, Baise, Guangxi Province, China; ^4^Department of Interventional Medicine, The Affiliated Hospital of Youjiang Medical University for Nationalities, Baise, Guangxi Province, China

## Abstract

Endothelial cells are heterogeneous, stemming from multiple organs, but there is still little known about the connection between the brain and kidney endothelial cells, especially in homeostasis. In this study, scRNA-seq results were obtained to compare genetic profiles and biological features of tissue-specific endothelial cells. On this basis, seven endothelial cell subpopulations were identified, two of which were upregulated genes in pathways related to stroke and/or depression, as characterized by neuroinflammation. This study revealed the similarities and distinctions between brain and kidney endothelial cells, providing baseline information needed to fully understand the relationship between renal diseases and neuroinflammation, such as stroke and depression.

## 1. Introduction

Endothelial cells play a crucial role not only in maintaining the biological functions of the brain and kidney but also in the development of renal and brain diseases, such as chronic kidney disease (CKD), stroke, and depression [1–4]. To date, it has been reported that several factors, such as VCAM-1, vWF, ICAM-1, P-selectin, and E-selectin [1, 2, 5, 6], related to endothelial cells are involved in either CKD or stroke/depression. Most of these are the common pathological factors for the tissue-specific diseases. Therefore, it is of practical significance to reveal the similarities and distinctions between brain and kidney endothelial cells.

In the present study, the scRNA-seq data collected from murine brains and kidneys in homeostasis were used to extract endothelial cells based on feature genes; genetic profiles were compared, and biological features were analyzed. Compared with kidney endothelial cells, two endothelial cell subpopulations were expressing a higher level of genes for three pathways closely linked to either stroke or depression, suggesting that these cells could be made susceptible to the disease by the upregulated expression of Ube2g1, Pdcd4, Fnbp4, Tollip, and Faf1.

With the use of a large-scale genetic profile, brain and kidney endothelial cells were compared and connected in this study, providing the baseline information required to explain the occurrence of neuroinflammation, especially stroke and depression, as observed in patients with renal disease.

## 2. Methods

### 2.1. Bioinformatic Analysis

The scRNA-seq results obtained from mouse biopsies were sourced from the NCBI GEO database. More specifically, data of healthy brains were accessed using GSE98816 [7], while the data of healthy kidneys were downloaded under the accession code GSE107585 [8]. For bioinformatic analysis, the *R* package Seurat was used to explore scRNA-seq data, while the *R* packages ggplot2 and Nebulosa were applied to draw violin plots, feature plots, and gene nebula maps. The *R* package Sctransform was adopted to eliminate variations between different platforms.

### 2.2. Functional Enrichment Analysis

*R* packages, including clusterProfiler, pathview, and Kyoto Encyclopedia of Genes and Genomes graph, were used to analyze and compare biological features of the enriched gene sets.

### 2.3. Laser Confocal Analysis

Kidney biopsies were obtained from five C57BL/6 mice. The tissue was embedded in O.C.T. compound and frozen in liquid nitrogen. The solid tissue was cut into multiple sections of 6 *μ*m thickness. After fixation in methanol at −20°C methanol for 10 min, the samples were blocked with phosphate-buffered saline (PBS)/0.5% BSA for 1 h at 4°C. Then, these samples were incubated with rat anti-mouse PECAM-1 (Invitrogen, #14-0311-85) overnight at 4°C. After being washed twice, they were incubated with A594 donkey anti-rat immunoglobulin G (Invitrogen, #A21209) and DAPI (Invitrogen, #D3571) for 1 h at 25°C. After washing twice with PBS, the sections were mounted for analysis using LEICA DEMI3000B.

## 3. Results

To minimize nonspecific classification, genes expressed in less than three cells were removed. Kidney biopsies were divided into 14 clusters (Figure 1(a)). For the identification of endothelial cells, there were four feature genes (Kdr, Pecam1, Cdh5, and Cd93) [7–9] used to determine the endothelial “location” on the feature plot (Figure 1(b)). Endothelial cells were concentrated in cluster 9. Laser confocal microscopy was performed to visualize the endothelial distribution in the kidney. With the staining of PECAM-1, which is an endothelial cell-specific marker, a blood vessel was identified around the glomerulus (Figure 1(c)). Notably, scRNA-seq experiments revealed that endothelial cells accounted for almost 3% of the total kidney (Figure 1(d)), which is much higher than that measured by laser confocal microscopy (0.8%), indicating that the newly developed technique, scRNA-seq, is far more sensitive than traditional microscopy.

Brain scRNA-seq experiments were performed using FACS-sorted endothelial cells, and the purity was verified [7]. For comparison between brain and kidney endothelial cells, the relevant data were integrated and subcategorized into seven subpopulations (Figure 2(a)). Specifically, the seven endothelial cell subpopulations were named by the seven genes expressed preferentially in different subclusters, including EC (B2m), EC (Ptn), EC (Sulf2), EC (Sncg), EC (Mapt), EC (Rpl38), and EC (Col6a1) (Figures 2(a) and 2(b)). To further examine the difference between these seven endothelial cell subpopulations, expression levels of the top 10 genes from each subpopulation were detailed in a heat map (Figure 2(c)). Each subpopulation demonstrated a specific genetic “fingerprint,” indicating the specific biological/pathological features of each subpopulation. To further compare the cellularity of endothelial cell subpopulations between the brain and kidney, a split-UMAP was used, and the frequencies were calculated according to scRAN-seq (Figures 2(d) and 2(e)). As shown in the stacked bar plot, four subpopulations were much “higher” in the brain than in the kidney, namely, EC (Ptn), EC (Mbpt), EC (Rpl38), and EC (Col6a1). It is suggested that these four subpopulations play a critical role in maintaining the vascularity of brain vessels, and that they could be more important to the development of brain diseases, such as stroke and depression. However, because of the limited number of cells in the subpopulation EC (Mbpt) and EC (Rpl38), these two subpopulations were removed from further analysis to avoid type II errors in statistics [10].

According to the Venn-pie chart, these two subpopulations, EC (Ptn) and EC (Col6a1), shared more than 85% of all differentially expressed genes (DEGs; brain vs. kidney) (Figure 3(a)), suggesting the similarity of their biological features in homeostasis and their potential to play similar roles in the development of brain diseases. To visualize the distribution of the “most significant” DEGs (log2 | FC | >1 and *p* < 0.05), the DEGs (Supplementary Figure 1 and 2) were marked in volcano plots (Figure 3(b)). Unexpectedly, nearly all of those “most significant” DEGs were concentrated in the upright section (upregulated DEGs), implying that these genes could play a more significant role in maintaining the homeostasis of the brain endothelium. To determine the expression levels of these DEGs, feature plots were used to reveal the pattern and level of expression of 10 randomly selected genes (Figure 3(c), Supplementary Figure 3), including Col6a1, Tnfrsf22, Abi3bp, Col6a3, Rhbg, H2-DMb2, Cdca8, Serpina3n, and Gfod1. These five genes were expressed at a much higher level in brain endothelial cells than in kidney endothelial cells.

When the DEGs derived from endothelial cell subpopulations, EC (Ptn) and EC (Cold6a1), were subjected to functional enrichment analysis, there were 3 critical pathways observed to be upregulated in brain endothelial cells: nucleotide binding, nucleoplasm, and ATP binding (Figures 4(a) and 4(b)). Further analysis was conducted to show that these three pathways play an active role in the development of stroke and depression [11–14]. As identified through GSEA, four of them were upregulated in brain endothelial subpopulations (Figure 4(c)). Furthermore, two genes (Ube2g1 and Pdcd4) were found to play a crucial role in the development of stroke [15, 16], and three genes (Fnbp4, Tollip, and Faf1) were found to be significant contributors to depression [17–19].

## 4. Discussion

With the assistance of scRNA-seq, extensive studies have been conducted to explore the heterogeneity of endothelial cells [7, 20] in the brain, lungs, and heart, thus improving our understanding of the biological and pathological features of endothelial cells. As for the similarities and distinctions between brain and kidney endothelial cells, there are still no studies focusing on the comparison between them through a large-scale genetic profile, even though they can be connected by sharing some common genes in homeostasis and inflammation.

Since it is widely known that pathology develops from homeostasis, detailing the connections of endothelial cells in the brain and kidney in homeostasis would contribute to improving our understanding of neuroinflammation, such as stroke and depression, as frequently observed in CKD patients. Pathological examinations can help reveal abnormal changes in both the brain and kidney endothelium in a significant proportion of patients with CKD [21].

In this study, we analyzed brain- and kidney-specific endothelial cells in homeostasis on a large-scale genetic profile. In this process, the endothelial cells in both organs were found to be highly heterogeneous, indicating their distinctive biological and pathological functions, which is consistent with previous reports [20]. Furthermore, two of them were found to be more closely linked to brain diseases, as evidenced by the upregulated expression of genes in three pathways, nucleotide binding, nucleoplasm, and ATP binding, all of which have been reported to be crucial for the development of stroke and depression [12–14]. These two endothelial cell subpopulations may be susceptible to disease. Notably, a significant proportion of patients with CKD develop either stroke or depression [22, 23]. This study has the potential to account for the observation that patients with CKD exhibit either stroke or depression.

In this study, two endothelial cell subpopulations were identified which could be essential for the development of neuroinflammation, stroke, and depression, from renal diseases. Moreover, there were 3 pathways identified as potential therapeutic targets to prevent brain dysfunction in patients with renal diseases.

## Figures and Tables

**Figure 1:** Identification of kidney endothelial cells. (a) UMAP plot shows 14 cell clusters in kidney. Cells in the red box are endothelial cells. (b) Feature plot shows the expression and distribution of 4 feature genes carried by endothelial cells. (c) Laser confocal microscopy reveals the phenotype of endothelial cells in kidney. (d) The comparison of endothelial cell frequency as analyzed by scRNA-seq and laser confocal microscopy.

**Figure 2:** Integrate analysis reveals endothelial cell heterogeneity. (a) UMAP plot shows the integrated analysis of brain and kidney endothelial cells, with 7 subpopulations classified: EC (B2M), EC (Ptn), EC (Sulf2), EC (Sncg), EC (Mapt), EC (Rpl38), and EC (Col6a1). (b) Violin plots show the expression level of 7 feature genes as identified from 7 endothelial cell subpopulations, namely, B2M, Ptn, Sulf2, Sncg, Mapt, Rpl38, and Col6a1. (c) Heat map shows the distinction between top 10 genes expressed in each endothelial cell subpopulation. (d) Split UMAPs show the comparison between endothelial cell subpopulations in the brain and kidney. (e) Stacked bar plot shows the comparison between endothelial cell subpopulations in brain and kidney.

**Figure 3:** Brain EC (B2M) and EC (Col6a1) exhibited upregulated genes related to stroke and depression. (a) Venn-pie chart shows the DEGs shared between EC (Ptn) and EC (Col6a1) and brain EC/kidney EC. (b) Volcano plots show the distribution of DEGs in EC (Ptn) and EC (Col6a1), respectively. Only log_2_FC > 0 and *p* < 0.05 are indicated by the plots. (c) Split feature plot shows the distribution and comparison of stroke and depression related genes in brain and kidney endothelial cells.

**Figure 4:** Brain EC (B2M) and EC(Col6a1) possess tumor/cancer-related pathways. (a) Dot plots show the enriched GO signaling pathways of the EC (Ptn) and EC (Col6a1), brain vs. kidney. (b) Gene-concept-network analysis of EC (Ptn) and EC (Col6a1), brain vs. kidney. (c) GSEA analysis reveals the upregulated or downregulated DEGs in the pathways (brain vs. kidney).

## Data Availability

The datasets and code created or analyzed in this study can be obtained from the corresponding author upon legitimate request.

## Supplementary Materials

Supplementary 1 Supplementary Figure 1: list of DEGs calculated from EC (Ptn).

Supplementary 2 Supplementary Figure 2: list of DEGs calculated from EC (Col6a1).

Supplementary 3 Supplementary Figure 3: comparison of the expression level of ten selected genes between brain and kidney endothelial cells. The *y*-axis is the relative expression level; *x*-axis is the identify of EC subpopulations: “0” refers EC (B2m), “1” refers “EC(Ptn),” 2 refers “EC(Sulf2)” 3 refers “EC(Sncg)” 4 refers “EC(Mapt),” 5 refers “EC(Rpl38),” and 6 refers “EC(Col6a1).”
